The article "Intelligent Network Teaching of Product Design Specialty Based on Video Image Processing" was retracted in 2023. Reasons: signs of a paper mill; suspected computer-generated content; unreliable results or conclusions; lack of ethics approval or compliance.

# Intelligent Network Teaching of Product Design Specialty Based on Video Image Processing

**DOI:** 10.1155/2022/6448995

**Published:** 2022-08-31

**Authors:** Zhimin Gao, Seungjin Lee

**Affiliations:** ^1^College of Fine Arts and Design, Huaihua University, Huaihua, 418000 Hunan, China; ^2^Graduate School of Education, Sehan University, Jeollanam-do 58447, Republic of Korea

## Abstract

The product design major was formally established in 2011 and has been an important part of Chinese art education since then. At the same time, it has laid a solid foundation for the development of China's higher education. Therefore, the product design major occupies an important position in China's higher education and plays an irreplaceable role in cultivating industrial design talents for the country. With the continuous development and progress of national education, the teaching of product design is also constantly innovating, in order to better improve the teaching effect of product design and cultivate more product design professionals for the country. The purpose of this paper is to study the teaching of product design major based on intelligent network teaching, establish an intelligent network teaching system, and carry out intelligent network teaching experiment of product design major based on this system. The experiment concluded that the overall satisfaction of the students majoring in product design on the intelligent network teaching reached 82%, and the intelligent network teaching mode also increased the outstanding performance rate of the students majoring in product design by 30%.

## 1. Introduction

The product design major is an art design major formally established in China in 2011. The education and training goal of product design major are to cultivate talents with strong sense of responsibility, advanced esthetic judgment, and systematic professional knowledge, and cultivate high-level composite art design application talents who can perfectly master the corresponding design thinking, communication, and management skills; can engage in research and development related to design and development; and can adapt to the needs of China's socialist modernization development. Over the years, the design talents trained by the product design professional education are mainly engaged in product design and have made great contributions to product design work in all walks of life in China. It can be seen that the product design major occupies an important position in China's professional education with the great progress of contemporary Chinese education, and the teaching of product design has also undergone significant changes and development. The progress and development of the product design profession can not only cultivate more outstanding product design professionals for the country, thereby promoting the development of the national economy, but also enable the country's education, especially higher education, to move towards a more brilliant future. The innovation and development of the teaching of product design must be inseparable from the support of certain science and technology. Intelligent network teaching refers to an advanced teaching mode that uses multimedia and intelligent network technology to assist teaching and achieve teaching goals under the guidance of certain teaching theories and ideas. This paper mainly conducts teaching research on product design based on intelligent network teaching.

The research innovations of this paper are as follows: (1) Combined with intelligent network teaching, this paper explores the teaching mode and method innovation of product design major. (2) In this paper, an intelligent networked teaching system is designed in combination with the intelligent network mapping algorithm, and based on the system, the teaching experiment of product design specialty is carried out, and effective experimental conclusions are drawn. (3) Compared with other researches on intelligent teaching, intelligent network teaching makes use of the Internet technology and the Internet, so that teaching work can be completed in different time and space.

## 2. Related Work

There has been a lot of research on intelligent teaching in academia. Among them, Chen S mainly studies piano teaching based on intelligent network teaching. He established an intelligent network piano teaching model and proved the effectiveness of the model to improve the effect of piano teaching through experiments [1]. Wu L's research first discussed the concept of the student model of the intelligent network teaching system, and then established a student model of the intelligent network teaching system based on the Bayesian network, and carried out the application experiment of the model [2]. Jing W conducted in-depth research on the ontology-based intelligent network teaching system. In his research, he first introduced the relevant theoretical basis, including the concept and structure of the intelligent teaching system, and then described the design of the ontology-based network intelligent teaching system [3]. Wen H mainly studies the intelligent network teaching based on computer-aided instruction (CAI) and uses the computer network collaborative learning mode and network teaching function to study the intelligent English teaching system [4]. Wang P's research focuses on the application of intelligent network teaching in badminton teaching. Through experimental analysis, he proved that the intelligent network teaching mode has a significant effect on improving students' interest in learning, technical movements, and theoretical knowledge level in badminton teaching classes [5]. Fang C mainly studied the application value of intelligent network teaching to the quality evaluation technology of English online teaching, proposed a teaching quality evaluation model combined with intelligent network teaching, and verified the practical effect of the model through experiments [6]. Although the above research has introduced and analyzed intelligent network teaching, it has not been combined with video image processing technology for comprehensive research. This paper will make a comprehensive analysis of this.

The above researches are closely related to intelligent network teaching and undoubtedly can provide a lot of information related to intelligent network teaching for the research of this paper. However, these studies are not practical enough for the research of product design based on intelligent network teaching, and the research angle is relatively single, and the research process is also more complicated.

## 3. Intelligent Teaching Methods for Product Design Majors

### 3.1. Image Class Web Teaching

Image is a visual description or picture of an objective object, and image is a more common information carrier in human social activities. The basic functions of intelligent network teaching are mainly distance teaching. If divided into major categories, there are mainly five aspects: web interface, homework management, teaching materials and learning tools, campus social network, and group learning. Modern images are based on real scenes and people, even fictional mythical animals and computer-generated virtual images are based on real objective objects. The image is an objective existence that arises from the real objective world.

Information transmitted by image media is extremely efficient in the reception of online teaching information. The human brain has functional subdivisions in which the brain areas related to visual information processing dominate compared to other senses. The memory for the rich information conveyed by images is the strongest. Images are the most direct in the communication process. Compared to the obscurity of the textual symbol system, image information can break the barriers of language and text and is not limited to the level of education of the audience. Language and words are specific symbolic systems of meaning. For example, the word “wood” is read and written in different ways in different languages and phonetics. It is impossible to understand without special study. However, the symbolic meaning system of images is a common language symbol system that can be read and understood by all human cultures, which can express basic meanings and even spread certain values and ideologies through the most direct images. Through the symbolic meaning system of images, ideological and political education can break through the limitations of cultural environment.

Image information has a strong visual impact. Whether it is shopping on the Internet looking at pictures or advertising on TV, or various colorful information in real life, it is also stimulated by the visual senses of these rich images. Images and new media are getting closer and closer to our lives, bringing great convenience to modern society. Today's online teaching efforts should have a place in this colorful world. It can take advantage of the convenience of image information dissemination and the advantages in terms of presentation, especially the combination of new media and network, which makes the scope of dissemination unlimited and the colorful content of dissemination. If the combination of network teaching and new media image media can make the content and material of network teaching education richer, it can make the enhancement of the scope of network teaching audience and the weakening of time and space limitation.

The so-called network teaching, as the name implies, is to use intelligent network technologies such as wireless networks and 5G communication networks to carry out network teaching. It is an efficient teaching mode in which schools use computer networks as the main means to implement information-based online education for students, and it is also an important form of distance teaching. Compared with the traditional teaching mode, online teaching can better cultivate students' abilities of information acquisition, processing, analysis, innovation, utilization and communication [7]. The network teaching mode is shown in Figure 1.

Compared with traditional education, online teaching has the following characteristics:

1. The teaching process has gradually changed from “teaching” to “learning”: teachers are no longer the main source of information, and students can actively obtain information through various channels
2. It realizes learner-centered personalized teaching. Network teaching has changed the traditional teaching mode of teacher-centered, classroom-centered and book-centered, and realized individualized teaching centered on students
3. It improves the learning efficiency of students. Through the use of multimedia technology, online teaching integrates video, audio, text, charts, and images, and presents the teaching content in front of students in a three-dimensional form, so that students can obtain information from all directions and angles, thus improving their learning interest and learning efficiency [8]

In addition, the interactive network technology in network teaching also realizes personalized learning. It can design the students' actual learning process, learning methods, and modes according to the actual situation of the students, thereby greatly improving the teaching efficiency and improving the teaching effect [9, 10]. The intelligent online teaching system is not only a function of distance teaching, but also includes class testing, while the constructivist learning theory has high requirements for learning testing, and the intelligent online teaching system just includes the learning test function.

### 3.2. Intelligent Network Teaching

Intelligent network teaching refers to an innovative modern teaching mode that applies advanced technologies such as intelligent communication technology, wireless broadband network technology, multimedia technology, and Internet of Things to assist teaching on the basis of traditional teaching methods, so as to efficiently achieve teaching goals. Intelligent network teaching adds intelligent elements to the teaching system through intelligent network and communication technology, making the entire teaching process more intelligent, and the teaching content presented is more diverse, intuitive, and visualized. And it can better meet the different requirements of learners to achieve personalized teaching, which greatly improves the teaching efficiency [11, 12]. The intelligent network teaching technology architecture is shown in Figure 2.The whole architecture diagram includes four parts: communication technology, intelligent network technology, multimedia technology, and students and teachers. The basic principle is that teachers use intelligent network technology, multimedia technology, and communication technology to teach students remotely.

Compared with traditional online teaching, intelligent online teaching has the following advantages:

1. It provides a virtual learning environment

Intelligent network teaching uses multimedia technology and virtual reality technology to create a realistic virtual environment for students to solve problems caused by material resources, financial resources, or time and space constraints. It can be seen that intelligent network teaching just makes up for the shortcomings of traditional network teaching in terms of interaction [13, 14].

(2) It provides personalized teaching services

Intelligent network teaching can provide students with personalized learning services, can meet the different needs of different learners, and then realize teaching according to their aptitude. By adopting the method of collective lesson preparation, the goal of optimizing the teaching content and improving the teaching level of teachers can be achieved. In intelligent network teaching, students are more subjective, and they can independently arrange their learning plans, freely decide their learning pace, and independently choose their learning time and place according to their actual situation [15].

(3) Intelligent teaching management

One of the most important tasks of higher education is teaching management. Therefore, establishing a scientific teaching quality assurance, evaluation, and recording system and implementing effective control over the teaching process are of great positive significance to the development of higher education. Intelligent network teaching can supervise the entire learning process of students, and can monitor the teaching process in real time, making teaching quality control more and more simple and intelligent [16].

### 3.3. Intelligent Network Mapping Algorithm

#### 3.3.1. Parameter and Variable Design

Due to the network installation environment, link failure, and natural disasters, it is necessary to ensure that the optical network can still guarantee the ability to send and receive services even when it suffers a certain degree of damage or failure. Therefore, while service requests are received and routes, wavelengths, and optical data units are allocated, the algorithm reserves a certain resource for protection routes. The protection route and the service working route pass through a completely different link. According to actual needs, the algorithm is also divided into full route protection mode and partial route protection mode. The former occupies a sufficient amount of optical data units, and when a fault occurs, the business can be directly converted from the working route to the protection route for transmission. The latter occupies a reduced-order optical data unit. When a fault occurs, the protection route can provide basic data and partial information of the service, which can assist in judging and determining the fault location [17, 18].

To sum up, the intelligent network algorithm should add the parameters shown in Table 1.

Similar to the working route, in the protection route, it is still necessary to allocate an appropriate optical data unit as a bearer for each service, denoted as *P* = *ϑ*(*k*)∗*k*. Among them, the route protection coefficient *ϑ*(*k*) can be expressed by the following formula:

(1) $$\begin{array}{c} \vartheta \left(k=1\right)=\left\{1k\right\}, \end{array}$$

And

(2) $$\begin{array}{c} \vartheta \left(\text{k}=2\right)=\left\{1,\frac{1}{2}\text{k}\right\}. \end{array}$$

That is, when *ϑ*(*k*) is always 1, it means that the algorithm is in the full route protection state, and when the link of the working route fails, it directly switches to the protection route for transmission. On the contrary, it is a partial route protection state, and all services are transmitted in the protection route by using reduced-order optical data units.

The service establishment situation in the protection route is represented by parameter *p*_*t*_. When the value of parameter *p*_*t*_ is 1, it means that the protection route is successfully established, and when it is 0, it means that the network is congested or the service establishment fails.

#### 3.3.2. Objective Function and Constraints

Similar to the algorithm of unprotected routing, in order to achieve the simultaneous equal distribution of information services and protection data for each link in the optical transmission network, the objective function of the algorithm with routing protection function is

(3) $$\begin{array}{c} \min\;R=S. \end{array}$$

The blocking rate in the objective function refers to the probability that a connection request is rejected, which can also be called the maximum number of connection requests. This objective function measures the maximum number of connection requests that can be carried in the network under the condition of a certain network capacity, namely

(4) $$\begin{array}{c} \min Z=\frac{\left|k\right|-\sum_{k}R}{\left|k\right|}. \end{array}$$

The network load measurement is the utilization rate of wavelengths in the network, and *m* represents the number of optical fiber links in the network, then

(5) $$\begin{array}{c} \min Z_{m}=\underset{k}{\sum }\frac{\text{ke}}{m}. \end{array}$$

Constraints in the intelligent network mapping algorithm refer to constraints on service routing and wavelength allocation based on the network structure itself.

First, let us look at the constraints of wavelength allocation: Services must meet the wavelength consistency principle during wavelength allocation. That is to say, a service can only occupy one wavelength in the network. If the connection request *k* is established, then, *k* needs to be allocated the same wavelength in the fiber link it passes through [19], as shown in the following formula:

(6) $$\begin{array}{c} \underset{\gamma }{\sum }x_{k}=\gamma k. \end{array}$$

The conflict constraint means that in a single-fiber system, each wavelength on the link cannot be occupied by two services at the same time; that is, different services on the same fiber have different wavelengths:

(7) $$\begin{array}{c} \underset{k}{\sum }x_{\text{ke}}=x^{\gamma }. \end{array}$$

On any link, the sum of the bandwidth occupied by all services and protection data transmitted on each available wavelength must be less than the maximum allocatable bandwidth of the available wavelength:

(8) $$\begin{array}{c} \underset{t}{\sum }\left[X_{t}\left(e,\gamma ,k\right)\right]. \end{array}$$

When assigning a protection route for a service, each link passing through should provide the same wavelength and the same bearer format:

(9) $$\begin{array}{c} \underset{e}{\sum }p_{t}\left(e,\gamma ,p\right)=\underset{e}{\sum }p_{t}\left(k\right). \end{array}$$

When the protection route of a service is transmitted through link *e*, the protection data can only occupy one wavelength, that is, only a single bearer format:

(10) $$\begin{array}{c} \underset{\gamma }{\sum }p_{t}\left(e,\gamma \right)=p_{t}\left(e\right),e\in E. \end{array}$$

The same as the working route, the protection route still needs to prevent the closed-loop phenomenon at the passing nodes, so the following constraints are imposed on the nodes that the protection route passes through

(11) $$\begin{array}{c} \underset{eE\left(v_{t}\right)}{\sum }P_{t}\left(e\right)=P_{t};t\in T, \end{array}$$

as well as

(12) $$\begin{array}{c} \underset{\text{ed}}{\sum }p_{t}\left(e\right)\leq 2P_{t}, \end{array}$$

And

(13) $$\begin{array}{c} \underset{e}{\sum }p_{t}\left(e^{\prime }\right)\geq p_{t}\left(e\right). \end{array}$$

In the algorithm for adding protection routes, the most important thing is the “avoidance principle” of working routes and protection routes; that is, they do not pass through the same link:

(14) $$\begin{array}{c} \underset{\gamma }{\sum }\underset{k}{\sum }p_{t}\left(e,\gamma ,k\right)+p_{t}k\leq 1, \end{array}$$

In the intelligent network mapping algorithm with protection routing function, the sum *R*_*e*_ of the bandwidth occupied by all services on the link *e* needs to consider the bandwidth occupied by the protection service. However, the constraint condition of the highest link utilization value *S* in all links does not change, and *R*_*e*_ can be written as

(15) $$\begin{array}{c} R_{e}=\underset{t}{\sum }\underset{k}{\sum }X_{t}\left(e,t,k\right);e\in E. \end{array}$$

The flow of the entire intelligent network mapping algorithm can be shown in Figure 3.

## 4. Intelligent Network Teaching Experiment of Product Design Major

### 4.1. Experimental Design

The main methods and steps of this product design professional intelligent network teaching experiment are as follows. Firstly, an intelligent network teaching system is established based on the intelligent network mapping algorithm, and then, the intelligent network teaching experiment of product design major is carried out based on the system. The purpose is to test the effect of the intelligent networked teaching system applied in the teaching of product design specialty. The experimental objects involved in the experiment are 30 students from class 1 of product design major in a university in Hangzhou. After the intelligent online teaching for these 30 students majoring in product design, they were tested for their satisfaction and teaching effect on this intelligent online teaching. After the test, according to the test results, judge the effect of intelligent network teaching of product design specialty based on the intelligent network teaching system designed in this paper.

The intelligent network teaching system designed in this experiment combined with the intelligent network mapping algorithm is shown in Figure 4.

The main contents of intelligent network teaching of product design major in this experiment are shown in Table 2.

### 4.2. Satisfaction Test of Intelligent Network Teaching

After the preliminary intelligent network teaching for the students in this class is over, this experiment tests the students' satisfaction with this intelligent network teaching. This satisfaction test mainly includes two aspects of students' satisfaction with the presentation of learning content and the organization of learning content. Among them, the test results of students' presentation of learning content are shown in Figure 5.

As can be seen from Figure 5, in this intelligent network teaching of product design major, a total of 13 students felt that the learning content of intelligent network teaching was more vivid, 10 students felt that the content was average, and 7 students felt that the learning content was effective and boring. As for the understanding of the presented learning content, a total of 16 students found it easy to understand, 9 students found it basically understandable, and only 5 students found it difficult to understand. To sum up, among the 30 students in this class, a total of 23 students were satisfied with the presentation of the learning content of this intelligent online teaching of product design, and the satisfaction rate reached 77%.

The test results of students' satisfaction with the learning content organization of this intelligent network teaching are shown in Figure 6.

As can be seen from Figure 6, in this intelligent network teaching experiment of product design major, a total of 25 students are basically satisfied with the organizational effect of learning content, and 26 students thought that the learning structure was less difficult to sort out. This shows that a total of 26 students are quite satisfied with the learning content organization of this intelligent network teaching, and the satisfaction rate has reached 86%.

Based on the analysis of the results in Figures 5 and 6, the overall satisfaction rate of the students participating in this intelligent network teaching of product design reaches 82%.

### 4.3. Test of the Effect of Intelligent Network Teaching

Next is the last step of this experiment, namely, test the teaching effect of this product design major intelligent network teaching. The test mainly obtains the results by judging the changes of students' learning efficiency and academic performance in intelligent network teaching.

First, in the process of this intelligent networked teaching, the test results of the changes in the learning efficiency of the participating students are shown in Figure 7.

As can be seen from Figure 7, in this intelligent network teaching, a total of 27 students out of the 30 students in this class have reduced their understanding time for the content they have learned by 1 hour or more. A total of 25 students saw a reduction of 0.5 hours or more in the consolidation of learning content. This shows that in this intelligent network teaching, the learning efficiency of most of the students in this class has been significantly improved.

The changes in the academic performance of the participating students are shown in Figure 8.

As can be seen from Figure 8, before the intelligent network teaching, the excellent rate of the students in this class in the midterm exam was 26%. After the intelligent network teaching, the excellent rate of the final exam results of the students in this class reached 56%. From this, it can be seen that the product design professional teaching based on intelligent network teaching has increased the student's outstanding performance rate by 30%.

To sum up, the conclusion of this paper based on the teaching experiment of product design major based on intelligent network teaching is that the overall satisfaction of product design majors on intelligent network teaching has reached 82%. The intelligent network-based teaching model has also increased the outstanding rate of product design students by 30%. The experimental conclusion of this paper fully shows that the product design professional teaching based on intelligent network teaching has achieved good teaching effect, which has a certain effect on improving the learning interest and achievement of the students who transfer to product design.

## 5. Discussion

The product design major plays an irreplaceable role in cultivating design professionals for the country and promoting the country's modernization and development. With the development of national education, the teaching of product design is constantly changing and progressing. The progress of product design teaching has also benefited from the development of science and technology.

The development of science and technology has brought many advanced technologies that can provide some technical support for the teaching reform of product design, such as intelligent network teaching. Compared with traditional teaching methods, intelligent network teaching incorporates more intelligent factors, making the whole teaching process more intelligent, vivid, and personalized, greatly improving teaching efficiency and teaching effect. This paper mainly studies the teaching of product design specialty based on intelligent network teaching.

In order to achieve the research goal, this paper designs an intelligent networked teaching system, and based on this system, the intelligent networked teaching experiment of product design specialty is carried out. The experiment mainly tested the satisfaction and teaching effect of the participating students on this intelligent network teaching. After the test, it was found that the overall satisfaction of the students majoring in product design on the intelligent network teaching reached 82%, and after the intelligent network teaching, the excellent rate of the students majoring in product design increased by 30%. The experimental conclusion of this paper fully shows that intelligent network teaching has a certain effect on promoting the teaching effect of product professional design.

## 6. Conclusions

This article makes an in-depth discussion of intelligent network teaching based on the professional technology of product design based on video image processing. Through experimental analysis, the research conclusions drawn in this paper show that intelligent networked teaching can also play some positive roles in the teaching of product design majors, which can promote the development of product design majors. It can effectively improve the learning interest and academic performance of product design students. The research of this paper has a certain significance for promoting the application of intelligent network teaching in the teaching of product design and also has a certain reference value for promoting the education innovation and progress of product design. However, the research of this paper also has some shortcomings, as follows: The research angle of intelligent network teaching is not comprehensive enough, only 30 students are selected for satisfaction survey, and no survey is carried out on people in other occupations, such as students' parents and teachers who use intelligent network teaching to teach. It is hoped that it can be improved in future research to make more contributions to promoting the teaching development of product design profession.

## Figures and Tables

**Figure 1:** Network teaching mode.

**Figure 2:** Intelligent network teaching.

**Figure 3:** Intelligent network mapping algorithm flow.

**Figure 4:** Intelligent network teaching system.

**Figure 5:** Presentation satisfaction test results of learning content.

**Figure 6:** Organizational satisfaction test results for learning content.

**Figure 7:** Student's learning efficiency change test results.

**Figure 8:** Changes in students' academic performance before and after intelligent networked teaching.

**Table 1:** Parameters to be added to the intelligent network algorithm.

Parameter	Describe	Function
*P*	Order of assignable optical data units in protection routing	Indicates the proportion of services transmitted in the protection link
*ϑ*(*k*)	Route protection factor	Determine the route protection method
*P*(*t*)	Indicates the service establishment in the protection route	Clear business establishment

**Table 2:** Contents of intelligent online teaching for product design majors.

Course program number	Course title	Course content
1	Design concept	Basic theoretical knowledge about product design
2	Product structure principle	Structural principles of product design
3	Interaction design fundamentals	Human-computer interaction design related theory and operation knowledge

## Data Availability

Data sharing not applicable to this article as no datasets were generated or analyzed during the current study.
